The article "Perception of Edentulous Patients and Dental Professionals towards Care and Maintenance of Complete Denture Prostheses" was published in 2022. Journal: Biomed Res Int.

# Perception of Edentulous Patients and Dental Professionals towards Care and Maintenance of Complete Denture Prostheses

**DOI:** 10.1155/2022/4923686

**Published:** 2022-07-11

**Authors:** Meenal Nand, Masoud Mohammadnezhad

**Affiliations:** ^1^School of Dentistry and Oral Health, Fiji National University, Suva, Fiji; ^2^School of Public Health & Primary Health Care, Fiji National University, Suva, Fiji

## Abstract

**Methods:**

A descriptive qualitative study was conducted among 30 EDPs attending dental prosthetic clinics (DPCs) at the four centres in Fiji and 28 DPs at the four DPCs under purposive sampling. Semi-structured questionnaire with open-ended questions was used for in-depth interview (IDI) with EDPs via telephone and focus group discussion (FGD) with DPs virtually via Zoom. Participant responses were recorded and thematic analysis was used to manually analyze the verbatim transcripts.

**Results:**

Five themes were identified as perceptions of EDPs towards care and maintenance of CDP in Fiji: patient perceptions towards CDP, CDP care and maintenance, communication between DPs and EDPs, challenges faced in CDP, and management strategies to CDP care and maintenance. Seven themes were identified as perceptions of DPs: CDP guidelines, post-denture insertion advice, care and maintenance, challenges while treating EDPs, management strategies to challenges faced, communication and teamwork, and recommendations to improving quality of CDP delivery in Fiji.

**Conclusion:**

Patients' perception towards care and maintenance of CDP was low. It is highly recommended for EDPs to adhere to CDP advice given by DPs whilst for DPs, it had been recommended to provide written, oral, and visual forms of CDP care and maintenance advice to EDPs for effectiveness.

## 1. Introduction

Poor oral health denotes social as well as physiological impacts on an individual together with affecting the overall life experiences and the self-esteem [1]. Edentulism in simple terms is a state of being without any natural teeth in the oral cavity [1–3]. Edentulism is a significant public health problem globally due to its high prevalence which is >10% in individuals 50 years and older and related disability [2, 4–7]. The World Health Organization (WHO) databanks indicate that caries is still prevalent in the majority of countries internationally, with some reporting 100% incidence in their populations; severe periodontal disease is estimated to affect 5% to 20% of the population, and the estimated rate of complete edentulism ranges between 7% and 69% internationally [3, 8, 9].

Complete edentulism displays a huge impact on the oral function of an individual such as speech and mastication [1, 10, 11]. For an individual, it is difficult to live a life without having a set of teeth and this is where complete dentures come into play. Complete dentures are the current common mode of treatment for the completely edentulous patients (EDPs) in order to improve the health with the establishment of effective function [12, 13]. Complete denture therapy brings about impactful outcomes in relation to its aesthetics and maintenance requirements regardless of it being highly associated with lack of confidence and problems related with chewing [1, 10, 12, 14]. Perception of dental professionals (DPs) also plays a keen role in the care and maintenance of complete denture prostheses (CDP) of the EDPs. The category of DPs who are involved in denture production is the dentists who are involved in the clinical stages and the dental technicians who are involved in the laboratory phase where the actual CDP is constructed [15]. Every dentist knows that the complete dentures are a set of prostheses that an EDP will not get adjusted to just in a few days but takes considerable amount of time and patience to adjust and adapt to a new “bulky foreign element” in the oral cavity [16]. Managing medically compromised patients can be a difficulty but that does not stop a DP from serving the elderly and needy community [17, 18] when it comes to improving prosthetic healthcare service delivery for the people of Fiji. For an EDP, the DPs are the major source of information channel regarding CDP; therefore, it is highly crucial that a DP has a thorough knowledge about the CDP and its related procedures in the fabrication.

There has never been a prior study done on CDP where patients and DPs like the dentists and dental technicians' perceptions were studied. There are a few previous studies on complete denture wearers [17, 19, 20] that had been conducted where the complaints based on care and maintenance of dentures and challenges of EDPs were elaborated [21]. This limited availability of information for a country like Fiji warrants for further research to be undertaken in this area which is essential in the lives of both the EDPs and the DPs in terms of exploring the perception of the EDPs and DPs towards the extent of care and maintenance given to their CDP in Fiji.

To fill the knowledge gap that was identified and ignored in the society on edentulism, it was highly relevant to have open discussions with the EDPs and DPs regarding their perception which included their views, problems, and personal suggestions and recommendations of improvement in their CDP and its care and maintenance in Fiji [21]. This study aimed to explore the perception of the EDPs and DPs towards the care and maintenance given to their CDP in Fiji.

## 2. Material and Methods

### 2.1. Design and Setting

This qualitative study was conducted among EDPs attending dental prosthetic clinics at the four centres in Fiji via telephone and DPs based at those four dental prosthetic clinics virtually via Zoom from 1^st^ August 2021 to 1^st^ September 2021. This method of conducting research during the Coronavirus (COVID-19) pandemic was the most effective in exploring perspectives of participants in a qualitative study [22]. This study had been undertaken at the Fiji National University (FNU) Dental Clinic and the three divisional dental prosthetic clinics (DPCs) in Fiji, namely, Colonial War Memorial Hospital (CWMH), Lautoka Hospital, and Labasa Hospital DPCs. Considering that they were the only specialty facilities in Fiji offering CDP treatments for the study samples, the corresponding clinics were chosen for the study.

### 2.2. Sample and Sampling

All EDPs that were male and female CDP wearers, 18 years of age and older, self-identified Fijians who had visited the four clinics during the study period, patients who were well-oriented to time and place, and patients who had promptly complied with postoperative instructions for complete dentures were all included in the study. EDPs with partial denture, suffering from Temporomandibular Joint (TMJ) disorders, psychological defect, severely resorbed ridge based on clinical assessment, and who did not want to participate were excluded from the study. DPs who were dentists or dental technicians with at least 6 months experienced, all age groups, valid registration with Fiji Medical and Dental Council (FMDC), male and females, DPCs at FNU, CWMH, Lautoka, and Labasa Hospitals were included in the study while dental hygienist, dental therapists, dental interns, private practice dental practitioners, those who did not practice, or DPs who were not willing to participate were excluded from the study.

Purposive sampling was done for EDPs attending the DPCs at FNU, CWMH, Lautoka, and Labasa Hospital where 30 participants met the criteria and were interviewed over telephone based on data saturation. Homogenous purposive sampling was done for DPs who were based at the DPCs at FNU, CWMH, Lautoka, and Labasa Hospital where 28 participants met the criteria and 4 focus group discussions (FGDs) were conducted virtually via Zoom consisting of 5-10 members per group until data saturation was reached.

### 2.3. Data Collection Tools

Two sets of semi-structured questionnaire with open-ended questions were developed for the study for EDPs and DPs, respectively, which was based on the review of literature and the research questions of the study. For EDPs, there were 2 sections of the questionnaire with a total of 14 questions of which section 1 comprised of the demographic information of EDPs like age, gender, marital status, and employment with 6 questions while section 2 had 8 open-ended questions associated with the perceptions of EDPs towards the care and maintenance of CDP translated in English, Hindi, and I-Taukei languages.

For DPs, there were 2 sections of the questionnaire having a total of 14 questions of which section 1 comprised of the demographic information of DPs like age, gender, marital status, and employment with 6 questions which was collected individually prior to commencement of the FGD.  Section 2 had 8 open-ended questions associated with the perceptions of DPs towards the care and maintenance of CDP in English translation.

### 2.4. Study Procedure

For EDPs, contact information for potential EDPs was provided by the 4 DPCs in Fiji who were later contacted via telephone call to request for their participation in their preferred language. The EDPs verbally agreed to participate after the consent form had been fully read to them over the phone prior to the start of the interview once they had a complete understanding of the procedure as explained to them in the information sheet. The verbally agreed consents by EDPs were recorded and compiled for the researcher's reference. The duration of in-depth interview (IDI) was 30-35 minutes. Each interview which was conducted by the researcher began with an introduction to the EDP which explained the purpose and conveyed the relevance of contribution to this study where all contributions were highly valued and remained confidential, and the interview was digitally recorded [23].

For DPs, potential DPs were initially sought by contacting the managers of the facility via email who were the principal dental officers of CWMH, Lautoka, and Labasa Hospital and the Head of School (HOS) of School of Dentistry and Oral Health (SDOH) to request for their participation virtually via Zoom one week before the commencement of the study. Information sheets were read to the DPs over Zoom regarding the details of the study in English medium for appropriate understanding. Once the DPs were fully aware of the process that was informed to them virtually from the information sheet, they gave their approval for participation by electronically signing the consent form which was emailed to them to be reverted prior to participation in the FGD forum. The researcher was the moderator for the FGDs. The duration for FGD was approximately 60 minutes.

Each FGD began with an introduction to explain the purpose and ground rules where opinions of every member of the group will be respected, listening to every member of the group, not to interrupt the members of the group while they were expressing their views and maintaining the FGD as highly confidential where whatever was discussed in the room shall remain in the room. Furthermore, conveying the importance of contribution to the study whereby all contributions were valued and remained confidential, and the session was digitally recorded [24].

### 2.5. Data Management and Analysis

The FGDs and interview's entirety were both transcribed into a Word document. Transcription was done verbatim where every single word was written down, including the pauses and the expressions of emotions such as laughter, stuttering, and hesitations such as “uh” and “ummm.” [25] The principal researcher completed transcription on the same day of the IDI and FGD. Transcriptions were reviewed repeatedly to remove all forms of identifiers from the data. The data was de-identified during transcription, and quotes were presented anonymously. In addition to that, listening to verbal cues and slight inflections in the participants' tone of voice was essential as it provided additional insight to the interview that was conducted [26]. Each interview and discussion with participants was assigned a code. Hard copies and electronic folders were created where all the information relating to the study and the participants were stored. Recordings were done separately from others and were labelled as per specific code. In each hard copy and electronic file, a division for each participant was created and stored.

Thematic analysis was conducted manually for encoding qualitative information and identification of themes or patterns, subthemes, and codes found in information that at minimum described and organized the maximum perceived characteristics of the phenomenon and probable observations [27]. The themes and subthemes which were identified were checked by the principal supervisor. The five steps involved in the analysis process were read and re-read of transcriptions to get general views, found repeated quotes from the extract, merged the quotes, merging of 2-3 subthemes into one, and used quotations.

### 2.6. Study Rigor

Four criteria fitting the study on its trustworthiness were transferability, credibility, dependability, and confirmability [28]. To ensure transferability, purposive sampling was adopted and the IDI was conducted until data saturation was reached. For credibility, participants were contacted and advised on the study before receiving approval for IDI and FGD, respectively; IDIs and FGDs were digitally recorded with same-day transcription performed by researcher and were thoroughly discussed with co-researcher at every stage. For dependability, IDI questions were same for all EDPs while FGD questions were same for all DPs which was initiated and executed through thorough systematic research of existing literatures; all data were coded and checked by co-researcher and transcriptions were re-read and noted to correct all errors. For confirmability, triangulation of data was adopted where EDPs had IDI while DPs had FGD conducted together with conceptual triangulation in exploring the qualitative data through frameworks in the study.

### 2.7. Ethical Considerations

Ethics approval was received from College Health Research Ethics Committee (CHREC). Facility approvals were received from the Head of SDOH for Fiji National University (FNU) Dental Clinic and the principal dental officers (PDOs) of the three Divisional Dental Hospitals.

The purpose and nature of the study were explained to the participant verbally via telephone calls for EDPs and virtually via Zoom for DPs by the researcher containing the information sheet which was in English version for DPs and in three versions that is, English, Hindi, and I-Taukei languages for the EDPs and voluntary informed consent obtained, respectively, as verbal for EDPs and written for DPs. They were also informed that their participation would be voluntary and information gathered in the interviews and discussions would be confidential. All soft copies of the information obtained from the IDIs and FGDs had been kept secured in the password-protected USB flash drive.

## 3. Results

Table 1 highlights the demographical characteristics of EDPs for IDI. Majority of participants were female (60%) from 60 to 70 yrs of age (60%). For ethnicity, majority of participants interviewed were Fijian of Indian Decent (FID) (87%) and were married (97%). Furthermore, based on employment status of participants, majority of participants were unemployed (93%) while the rest were employed (7%). Furthermore, on divisions, most participants were from central division since CWMH dental clinic and FNU dental clinic constituted to majority of participants (54%).

### 3.1. Themes Identified for EDPs

Five themes had emerged from thematic analysis: patient perceptions towards CDP, CDP care and maintenance, communication between DPs and EDPs, challenges faced in CDP, and management strategies to CDP care and maintenance.  Table 2 summarizes the themes and subthemes analyzed in the study. A participant number was assigned to each EDP such as P1, P2,... Gender for EDPs was coded as M or F and ethnicity of EDPs was as I-Taukei (IT) or Fijian of Indian decent (FID).

#### 3.1.1. Theme 1: Patient Perceptions towards CDP

EDPs had stated various details of information on their perceptions on CDP they had such as knowledge on CDP, positive patient attitude vs negative patient attitude, and experiences of EDPs in wearing CDP.

*(1) Knowledge on CDP*. The participants had a fair knowledge about CDP that they had.

*About this teeth, I made these teeth to help me eat food properly including the hard food but I also eat soft food … and even feel looseness of the denture.* (P5, 57-year-old, M, FID)

Some EDPs were well advised by DPs when they received CDP on “what to do and what not to.”

*I was told to make sure I don't eat anything that is very hot for my dentures…while eating food.* (P18, 65-year-old, M, FID)

*(2) Positive vs Negative Attitude*. Some patients were so impressed with the quality of service being provided to them for their CDP that they wished to get new sets fabricated after using dentures for a long time.

*My view on these dentures are very good. I am thinking of getting another one made… for myself sometime soon.*(P30, 65-year-old, F, FID)

Some patients still did not feel satisfied with the CDP they received as they still face some problems with it which does not allow them to wear appropriately.

*I have been given a very nice set of dentures from the hospital. But, but I also face some problems wearing… I got it.* (P9, 70-year-old, M, FID)

*(3) CDP Wearing Experiences*. Majority of EDP gave good responses about their CDP prior to their previous dentures.

*When I wear people say I look nice,… and good.* (P1, 68-year-old, F, IT)

There were also a few EDPs who were not satisfied at all with the CDP that was fabricated for them.

*This denture is not good for me. I cannot … this denture.* (P25, 69-year-old, M, IT)

#### 3.1.2. Theme 2: CDP Care and Maintenance

Information on the methods for CDP cleaning and maintaining, common denture cleaning products, and CDP storage were comprehensively highlighted.

*(1) Methods for CDP Cleaning and Maintaining*. Vast number of EDPs had their own rules for cleaning dentures and ensured they performed on a daily basis.

*In the morning, I also occasionally use soap … and clean it.* (P7, 61-year-old, F, FID)

Some EDPs were advised by DPs that they should not apply Colgate on their dentures anytime as it will erode the acrylic teeth thus reducing its size.

*I use a brush and clean the dentures properly … not to use Colgate … size of my teeth on my dentures.* (P29, 53-year-old, M, FID)

*(2) Common Denture Cleaning Products*. A significant number of EDPs utilized denture cleaning material which is available at home.

*To clean I only use salt,… on my dentures to clean.* (P13, 71-year-old, F, IT)

Financially stable EDPs purchased denture cleaning medications from local pharmacies for cleaning and maintaining CDP.

*I got a medication from pharmacy, a tablet … overnight when I go to sleep.* (P29, 53-year-old, M, FID)

*(3) CDP Storage*. Majority of patients stated they stored their CDP appropriately in containers.

*I look after my teeth well. I clean them all the time … then store it in a container with lid.* (P5, 57-year-old, M, FID)

Few patients who do not have availability of good containers resorted to other modes of storing CDP.

*In the evenings, I take off my denture and put it in a jar of water and then … wash them properly.* (P19, 69-year-old, F, FID)

#### 3.1.3. Theme 3: Communication between DPs and EDPs

EDPs expressed their views on how DPs communicated with them from day one of CDP treatment process on CDP that was fabricated. Information on passive obedience and patient motivation and trust was presented, respectively.

*(1) Passive Obedience*. A number of patients personally put a lot of effort in wearing CDP.

*Well I am able to wear my denture … got the denture glue …with these dentures.* (P12, 52-year-old, F, FID)

EDPs agree that irrespective of the amount of assistance by CDP, it will not be like their natural teeth.

*My dentures are very good but then it's still not like the permanent teeth.* (P15, 64-year-old, F, FID)

*(2) Motivation and Trust*. Majority of patients were fully motivated to wear CDP.

*Oh yes, I am able to eat very well with this set of teeth … talk with everyone at home so well when I wear teeth.* (P3, 66-year-old, F, FID)

#### 3.1.4. Theme 4: Challenges Faced in CDP

EDPs encountered numerous challenges while wearing CDP. Challenges like lack of information, noncompliance of patients towards CDP wearing, reduction in QoL of the CDP patients, and financial barriers to CDP treatment costs on CDP were featured under this theme.

*(1) Lack of Information*. A couple of patients commented they had no information about CDP.

*I don't have much knowledge on this denture. Just how I clean … about this teeth.* (P12, 52-year-old, F, FID)

Participants stated that there was nothing explained by DPs about complete denture rehabilitation when attended dental clinic to make CDP.

*When I went to make my teeth they don't tell me anything … and make mine.* (P13, 71-year-old, F, IT)

*(2) Noncompliance*. A few patients found it very difficult to wear CDP.

*Because I get blisters by wearing the lower dentures…I do get headaches … try to work at home.* (P14, 69-year-old, F, FID)

Few participants mentioned they faced difficulty with eating and speaking when using CDP.

*First 2* days *I faced some difficulties … tried to eat … wearing the dentures.* (P18, 65-year-old, M, FID)

*(3) Reduction in QoL*. Patients with shallow ridges with lower loose dentures are unable to live normally with CDP.

*The small problem faced in my lower denture…does cause slight disturbance.* (P7, 61-year-old, F, FID)

EDPs also mentioned that loose dentures are of no help.

*The denture is slack so it disturbs me … it comes out of the mouth.* (P25, 69-year-old, M, IT)

*(4) Financial Barriers to CDP Treatment Cost*. The current cost of getting a denture is reasonable for many EDPs.

*I am a social welfare recipient … made for free*. (P28, 65-year-old, F, FID)

Few participants did not want to spend money going back to get dentures made as were not sure they would find the staffs.

*I did not spend money going for my review … in fixing my dentures.* (P30, 65-year-old, F, FID)

#### 3.1.5. Theme 5: Management Strategies to CDP Care and Maintenance

EDPs undertook management strategies to ensure care and maintenance of CDP are achieved. Motivation towards CDP hygiene, support from family members, and valuing engagement with DPs for reinforcement were mentioned under this theme.

*(1) Motivation towards Daily CDP Hygiene*. Most patients continued wearing CDP instead of going to the hospital after which they eventually got used to their prostheses.

*For the problems I had I …continued wearing my false teeth regularly … pain eventually went away.* (P2, 67-year-old, F, FID)

Some participants applied Bonjela and were able to manage the problem.

*One place which was hurting me … applied Bonjela … and its good now and i feel much better.* (P4, 64-year-old, F, FID)

*(2) Support from Family Members*. EDPs appreciated the support they got from families at home in improving their speech using CDP.

*I am very happy … talk very clearly with my grandchildren when I try to talk with them.* (P6, 74-year-old, F, FID)

Irrespective of immense family support, one participant expressed his unsatisfaction towards CDP.

*Eating time, when I try to eat cassava with my family, the denture is slack.* (P25, 69-year-old, M, IT)

*(3) Valuing Engagement with Dental Professionals for Reinforcement*. EDPs had appreciated a job well done by DPs for process they took them through in getting CDP.

*I thank all the staffs who are engaged in this denture making team…Due to them … using our dentures today.* (P6, 74-year-old, F, FID)

One participant mentioned that he is still not content with his CDP regardless of numerous visitations and advices received from DPs.

*From the advice…I am still not able to chew food like roti properly… comes out.* (P12, 52-year-old, F, FID)

Table 3 highlights the demographical characteristics of DPs for FGD. Majority of participants were female (82%) from 20 to 30 yrs of age (43%) and were FID (82%). Furthermore, most participants were classified as dental technicians (DTech) (57%). Most DPs were from government/public sector (79%) with majority from central division (57%).

### 3.2. Themes Identified for DPs

Seven themes emerged from thematic analysis: CDP guidelines, post-denture insertion advice, care and maintenance, challenges while treating EDPs, management strategies to challenges faced, communication and teamwork, and recommendations to improving quality of CDP delivery in Fiji.  Table 4 summarizes the themes and subthemes analyzed in the study. Each FGD was given FGD number like FGD1, FGD2,… The classification of DPs was coded as dental technicians (DTech) and dental officers (DO).

#### 3.2.1. Theme 1: CDP Guideline

DPs highlighted on CDP guidelines where areas like CDP fabrication guideline and CPGs and DPs knowledge on CDP were comprehensively discussed.

*(1) CDP Fabrication Guideline and CPG*. Majority of participants stated CDP fabrication procedures and dental CPGs need to be effectively followed to produce high-quality CDP.

*We need to follow CPG in order to achieve … best prostheses…to gain suction of those dentures.* (FGD 1, 45-year-old, DTech)

Most participants stated that procedures for CDP fabrication both from the clinic and dental laboratory need to be correctly followed.

*So I mean … primary impression gives us some basic foundation to build up our, our second impressions on…for processing.* (FGD 4, 33-year-old, DO)

*(2) DPs Knowledge on CDP*. Most DPs mentioned that CDP fabrication involves many stages.

*These dentures are made in many stages … to be nicely done so that final product is good.* (FGD 1, 40-year-old, DO)

All DPs stated the importance of planning each CDP treatment visit.

*There's about four to five visits required …for a complete denture prosthodontics.* (FGD 4, 33-year-old, DO)

#### 3.2.2. Theme 2: Post-Denture Insertion Advice

DPs discussed the post-denture insertion advices provided to EDPs once a CDP is given. Information on guide and instruction to CDP wearing and care and patient motivation had been highlighted here.

*(1) Guide and Instruction to CDP Wearing and Care*. One participant had reiterated on the importance of giving postoperative advice to the patients who receive CDP to help them in masticatory processes.

*It is important to give post-op advise to the patient … could help in maintaining it.* (FGD 1, 25-year-old, DO)

Another participant highlighted there are prosthetic postoperative care leaflets given to patients visited the government dental clinics for CDP.

*The post-operative leaflet consisting of post-op advise is given to the patients … by both clinician and technician.* (FGD 2, 54-year-old, DO)

*(2) Patient Motivation*. Participants expressed the need for motivating EDPs to continue wearing CDP.

*Motivating the patient is very important … so that they get used to the denture.* (FGD 1, 45-year-old, DTech)

DPs also mentioned that in order for EDPs to be motivated requires willingness coming from EDPs themselves.

*And if the willingness from the patients …the more comfortable, more adaptable it's going to be right.* (FGD 4, 43-year-old, DTech)

#### 3.2.3. Theme 3: CDP Care and Maintenance

DPs expressed views relating to care and maintenance of CDP where subthemes surfaced were on the do and dont's of CDP care and maintenance and home care remedies to CDP care and maintenance.

*(1) Do's and Dont's of CDP Care and Maintenance*. Participants mentioned that a few patients prefer to sleep at night wearing CDP.

*How to clean it,… some patients want to sleep with their denture full time.* (FGD 3, 31-year-old, DO)

Majority of DPs declared that process of denture maintenance does not just involve patient effort but also equal efforts from DPs ensuring EDPs adhere to guidance provided.

*The maintenance of complete denture, it involves both the patient, patient doing their part and as well as a clinician doing their own part as well.* (FGD 4, 35-year-old, DO)

*(2) Home Care Remedies to CDP Care and Maintenance*. One DP remarked on reminding patients throughout the denture making process on how these CDPs need to be kept clean to avoid any fungal build up.

*I usually tell patients throughout the denture making process towards good denture hygiene … Not just bacteria but fungal … denture stomatitis, things like that.* (FGD 3, 31-year-old, DO)

DPs also agreed to daily practicing of good denture habits to maintain their dentures effectively.

*Like denture cleaning with effective and non-abrasive cleaners and brush. Do not soak it in bleach.* (FGD 3, 25-year-old, DTech)

#### 3.2.4. Theme 4: Challenges While Treating EDPs

DPs emphasized on challenges faced while treating EDPs. Subthemes emerged were language barriers, patient noncompliance, and CDP comparison (comparing old dentures with new dentures and patient to patient denture comparison).

*(1) Language Barriers*. Most participants mentioned some EDPs specially from different ethnic backgrounds faced difficulties understanding English.

*If the patient doesn't understand our language, we try to call in an officer who speaks their language.* (FGD 1, 40-year-old, DO)

Some participants highlighted EDPs do not understand the dental terminologies.

*Most of the patients, they don't understand our terms,… explain things to them in their native language.* (FGD 2, 29-year-old, DO)

*(2) Patient Noncompliance*. Number of DPs mentioned that EDPs find difficulty speaking with CDP.

*Another problem is the patient sometimes find it difficult, I mean difficulty in speaking … front of the mirror and get used to it.* (FGD 1, 27-year-old, DO)

Participants highlighted on mixing and matching CDP by EDPs and wearing with comfort.

*Some of them they want to like mix and match their old denture with the new denture and wear it.* (FGD 3, 25-year-old, DTech)

*(3) CDP Comparison (Old CDP vs New CDP and Patient to Patient Comparison)*. DPs highlight EDPs are not accepting that old denture is different from new CDP that will improve mastication.

*They start comparing their dentures …patients have 2 sets of dentures so they start comparing … new set of dentures.* (FGD 1, 34-year-old, DTech)

Majority of participants experienced patients who continue wearing old set of teeth regardless of having a new set.

*Patients they normally … their old dentures, they still wear after getting a new pair of dentures* (FGD 3, 25-year-old, DTech)

#### 3.2.5. Theme 5: Management Strategies on Challenges Faced

DPs elaborated on management strategies on challenges faced. Theme and the subthemes that came up were modifying of CDP treatment and fabrication approach, addressing patient expectations from day 1 of treatment, promoting effective patient participation throughout treatment process, and incorporating verbal, written, and translated advice to EDPs.

*(1) Modifying CDP Treatment and Fabrication Approach*. Majority of DPs highlighted that especially, to meet CDP demand for aged patients, treatments are modified.

*For patients with existing dentures, what we do is we take secondary impression on their existing denture … to overcome that challenge.*(FGD 1, 45-year-old, DTech)

One participant shared that for loose dentures, adhesives can be utilized to ease the problem temporarily.

*I guess, for patients who don't have good denture stability due to atrophic ridge. They can use a denture adhesive.* (FGD 3, 31-year-old, DO)

*(2) Addressing of Patient Expectations from Day 1 of Treatment*. Participants also mentioned that EDP expectation needs to be addressed prior to commencement of CDP treatment.

*So that is very, very important as a clinician, from the onset, not from the day you tell the patient … means from day one.* (FGD 4, 35year-old, DO)

Majority of participants mentioned to allow EDPs to see reality of the situation from day 1 of CDP treatment.

*That expectation has to be made into reality in the first visit … to advise them.* (FGD 4, 33-year-old, DO)

*(3) Promote Effective Patient Participation throughout Treatment Process*. DPs practice this by using demonstrative models to EDPs explaining CDP treatment process.

*We try to keep models showing different heights of ridges … why their denture is more retentive.* (FGD 1, 34-year-old, DTech)

Rapport building is another method to keep EDPs engaged throughout CDP process.

*And I think rapport building is very important … if they like you.* (FGD 2, 24-year-old, DO)

*(4) Incorporating Verbal, Written, and Translated Advice to EDPs*. DPs noted that caregivers who usually accompany EDPs are not educated thus additional barrier in advising EDPs.

*The mental capacity … really old and they always like, they usually have a caregiver with them…and then the caregivers are not able to do the same for the patient as well.* (FGD 3, 31-year-old, DO)

DPs elaborated on importance of translators in dental clinics to ease the language barrier when communicating with EDPs.

*One more thing … translators that really helps as well … even during the stages of denture construction.* (FGD 4, 33-year-old, DO)

#### 3.2.6. Theme 6: Practice of Communication and Teamwork

DPs explained on practice of communication and teamwork in CDP care and maintenance. Subthemes highlighted were staff communication (dentist and dental technician) and triangle of communication and information sharing (dentist-dental technician and patient).

*(1) Staff Communication-Dentist and Dental Technician*. DPs mentioned that effective collaboration between dental officer and dental technician is an essence of a successful CDP treatment outcome.

*Very important as a dental officer is to work in collaboration with the technicians…it's always good to listen.* (FGD 1, 40-year-old, DO)

Effectiveness of communication between dental officers and dental technician throughout the CDP fabrication process was the highlight of the discussion.

*So it's very important that we as clinician, we need to communicate … outcome of the denture would be good.* (FGD 2, 24-year-old, DO)

*(2) Triangle of Communication and Information Sharing (Dentist-Dental Technician and Patient Communication)*. Majority of dental officers appreciate the role dental technicians play in fabricating high-quality CDP.

*When the technicians come and see patients and the case based on their expertise, the quality of prosthesis really goes up … during difficult times.* (FGD 1, 40-year-old, DO)

Participants agreed to undergo continuous communication throughout the treatment to keep EDP encouraged.

*I think it's the relationship that you have with your patient,… is really important.* (FGD 4, 50-year-old, DTech)

#### 3.2.7. Theme 7: Recommendations to Improving the Quality of CDP Delivery in Fiji

DPs stated recommendations to improving quality of CDP delivery in Fiji. Genuine subthemes generated were further education, standardizing workload, decentralization of dental prosthetic services, and increasing employability for DPs.

*(1) Further Education*. Further education for DPs in the area of dental prosthetics and dental technology will improve clinical and laboratory skills.

*I think training to be needed … can help with the patient management as a whole.* (FGD 2, 29-year-old, DO)

Participants commented on effectiveness of continuous professional development for improved CDP service delivery.

*It's just continuously improve your knowledge,… from my point of view.* (FGD 4, 50-year-old, DTech)

*(2) Standardizing Workload*. DPs indicated the need to standardize workload for DPs so quality output can be achieved.

*There shouldn't be a lot workload. If the workload increases…So targets should be realistic … prostheses that are more acceptable to the patients.* (FGD 1, 40-year-old, DO)

Majority of participants believe standardization of procedures will bring about harmonious CDP service delivery.

*And with dentures and like any other case, the more you do, the better you get. …you know there are people to assist us.* (FGD 4, 33-year-old, DO)

*(3) Decentralization of Dental Prosthetic Services*. Participants mentioned the need to open more dental prosthetic clinics in all divisions in Fiji to improve CDP delivery.

*Probably open up another lab … providing prosthetic services to the whole of Northern Division.* (FGD 1, 34-year-old, DTech)

Further comments on expanding dental prosthetic service delivery in the maritime region in Fiji.

*We need to look into opening more dental prosthetic not only at divisional level.* (FGD 3, 35-year-old, DO)

*(4) Increasing Employability for DPs*. Majority of participants mentioned due to huge CDP demand in Fiji, there is a need to create more employment for DPs.

*There is lot and just with one lab we are not able to cater the demand.* (FGD 1, 34-year-old, DTech)

Participants mentioned that increased employment for DPs means optimum participation in Public Health Awareness campaigns throughout Fiji.

*When it come to do with awareness… public to know about what is going on.* (FGD 3, 47-year-old, DTech)

## 4. Discussion

Perceptions of EDPs identified were patient perceptions, CDP care and maintenance, communication between DPs and EDPs, challenges faced in CDP, and management strategies to CDP care and maintenance.

Patient perception plays a vital role towards having an appropriate understanding on the care and maintenance of CDP in Fiji. From this study, it was revealed that EDPs have had adequate knowledge of the CDP that they received from the dental clinics to assist them in their daily lives through improving mastication, speech, and socialization as well as improving their appearance. Gupta, S. et al. revealed that 58.3% of the population have had positive attitude towards having CDP fabricated while 74.8% of the population had strongly agreed that oral hygiene maintenance for CDP is highly necessary [29].

CDP are cleaned and maintained mechanically and also chemically by EDPs in order to increase the longevity of the denture. Saha, A. et al. found out that rinsing CDP with water had been most commonly used method for cleaning and maintaining dentures [30] which was what that had been found in this study in relation to EDPs in Fiji context. Patients mentioned on storing CDP in a container where the dentures are immersed in water and covered with lid overnight. A literature by Verhaeghe, T.V. et al. found out that if dentures are not stored using denture tablets, then there should be wider considerations given to storing dentures dry as no changes in the dimensional stability of dentures were noted if stored dry for 8 hours [31].

This study showed that EDPs had a great trust on their DPs who had provided quality CDP which greatly correlated to Emami. E. et al., Marchini, L., and Cerruti-Kopplin, D. et al. stating numerous factors were involved in CDP care and maintenance like technique-related factors, DP-related factors, patient factors, personal, financial, social factors, and also health-related factors which triggered to enforce the sense of motivation and trust by the EDPs on their DP for quality CDP care services [32–34].

Some EDPs had reported that they had very less to no knowledge on the CDP they had received from their dentists on how to clean and maintain their CDP as well. Similar sentiments were highlighted by Nand M. and Mohammadnezhad M., Berteretche, M. V. et al., and Sjogren, P. et al. stating patients were not informed about CDP care and maintenance which led to lack of oral hygiene and poor perception of denture care in EDPs [21, 35, 36].

Family members played a vital role in keeping EDPs motivated towards wearing the CDP as well as effectively cleaning and maintaining it for the longevity which had been highlighted by Hsu, Y. J. et al. stating that there is involvement of family members of EDPs as well when they are visiting the dental clinics to support the CDP fabrication process and keep the EDP motivated in the treatment process [37].

Perceptions of DPs identified were CDP guidelines, post-denture insertion advice, care and maintenance, challenges while treating EDPs, management strategies to challenges faced, communication and teamwork, and recommendations to improving quality of CDP delivery in Fiji.

DPs had a thorough knowledge on CDP guidelines which involved the CPG and CDP fabrication guideline that had been enacted and utilized in Fiji by every DP. In addition, few of the participants had been part of the CDP guideline policy making process. The current enacted policy had not been a very detailed guideline urging a greater need for reviewing of the policy in order to keep in line with the updated knowledge and new developed technology in the area of Prosthetic Dentistry which the current DPs in the areas of dentistry are well versed with. The DPs which involved the dental officers and the dental technicians stated that both CPG and CDP policy guidelines need to be revised to suit the current context in Fiji regarding CDP service delivery relating to literature stating that DPs need to keep themselves updated and understands that at population level, CDP treatment service delivery varies and is changing whereby a great number of EDPs would still require CDP treatment [38, 39].

Post-denture insertion advice was appropriately delivered to EDPs by DPs to ensure adherence to postoperative care is maintained. On the contrary, Peracini, A. et al. and Curtis, S. et al. stated that EDPs did not receive proper denture cleaning instructions from their DPs [40, 41].

According to DPs, EDPs had been quite careless in taking care and maintenance of their CDP. DPs mentioned that most common form of denture cleaning and maintaining taken up by the EDPs in Fiji is using a brush to wash under running water being globally consistent with known literatures from Saha et al. (47%), Patel et al (58.3%), Dikbas (3.84%), Peracini et al. (3.7%), Azad et al. (22%), and Apratim et al. (31.3%) [30, 40, 42–45].

Understanding each other's language had been important for EDPs and the DPs. It has been found that some EDPs specially from different ethnic backgrounds faced difficulties understanding English. Pasad. A. K. et al. found out that patients usually felt more comfortable conveying their feelings, concerns, doubts, and fears regarding CDP treatment in their language, as reported by 429 (85.8%) patients considered that the DPs understanding their language are important for them [46].

A DP had stated that expectations of EDPs on their CDP can be challenging at times. This was consistent with the literature by Zou Y. and Zhan D. where it was found that DPs need to be fully aware of EDPs expectations before treatment and provide them with detailed introduction into the problem, which not only aims to explain the limitations and possibilities of CDP treatment per se but also assists the EDP to learn how to cope with the CDP [47].

All DPs had stated on having an effective collaboration between each other when treating EDPs particularly the collaboration between DOs and DTechs. This finding had been evident in a literature by Hatzikyriakos, A. et al. where it was stated that almost 30% of patients shade selection was performed by dental technicians in dental laboratories with the EDPs [48].

It has been found in the study that further education for DPs in the area of dental prosthetics and dental technology improved their clinical and laboratory skills on CDP fabrication through practice and attending CPD sessions benefitting the EDPs in Fiji. This finding is consistent with literature from Wieder, M. et al. and Clark R K F. et al. where it was found that lack of experience resulted in new graduates entering vocational training with little confidence in denture techniques and unable, sometimes unwilling, to undertake these procedures related to CDP [49, 50].

### 4.1. Limitations

The study included only EDPs and DPs. It would be ideal for future researchers to include partially dentate patients (PDP) and the dental hygienists (DH) who are also present and rostered with the DO during dental prosthetics at DPC. Due to COVID-19 restrictions, participation of the members from the two target groups was virtual via Zoom for DPs and via telephone call for EDPs. Due to COVID-19 restrictions, verbal consent was received from the EDPs after the information sheet and consent form was fully read out to them while the DPs had electronically signed the consent forms and were emailed back to the researcher. Data collection was timed based on participant availability because of the study's environment and participants' nature, and finally the education level of EDPs was not investigated under demographic characteristics of the study.

## 5. Conclusion

EDPs' perception on care and maintenance of CDP was moderate based on the post-denture insertion advices that were received which helped the EDPs in attaining a broader and better understanding of CDP and the level of expectations being held when undergoing CDP treatment in the dental clinics in Fiji. DPs perceptions on care and maintenance of CDP assisted in the provision of relevant as well as alarming information on the challenges faced with recommendations of improving CDP service delivery for the EDPs in Fiji. What EDPs and DPs require in order to have a clear perception about CDPs is the improvement in the quality of CDP and development of new CDP post-insertion guidelines which can be both adapted by DPs and elaborated effectively to EDPs for appropriateness. The DPs who are one of the groups of participants of this study are highly qualified and knowledgeable group of individuals in the area of dentistry. However, the larger goal of getting no complaints regarding CDP from EDPs is something which may be impossible as every individual has a different level of adaptation to its CDP. At the heart of many participant's concerns were if proper guidelines can be followed always in order to ensure appropriate denture care and maintenance advice is given to patients by the DPs and the DPs came up with effective recommendations on improving complete denture fabrication which would lead to improve in the quality of CDP as well as service delivery in Fiji.

## Figures and Tables

**Table 1:** Demographical characteristics of participating EDPs for IDI (*n* =30).

Characteristics		Frequency (*n*)	Percentage (%)
Gender	Male	12	40
	Female	18	60
Age groups	50-60 yrs	7	23
	60-70 yrs	18	60
	70-80 yrs	5	17
Ethnicity	I-Taukei	4	13
	Fijian of Indian decent	26	87
Marital status	Single	0	0
	Married	29	97
	Divorced	1	3
Employment status	Employed	2	7
	Domestic duties	28	93
Division	Northern	7	23
	Western	7	23
	Central	16	54

**Table 2:** Themes and subthemes identified from IDI analysis.

Themes	Subthemes
Patient perceptions towards CDP	Knowledge on CDP
	Positive vs negative attitude
	CDP wearing experiences
CDP care and maintenance	Method of CDP cleaning and maintaining
	Common denture cleaning products
	CDP storage
Communication between DPs and EDPs	Passive obedience
	Motivation and trust
Challenges faced in CDP	Lack of information
	Noncompliance
	Reduction on quality of life (QoL)
	Financial barriers on CDP treatment cost
Management strategies to CDP care and maintenance	Motivation towards daily CDP hygiene
	Support from family members
	Valuing engagement with dental professionals for reinforcement

**Table 3:** Demographical characteristics of participating DPs for FGD (*n* =28).

Characteristics		Frequency (*n*)	Percentage (%)
Gender	Male	5	18
	Female	23	82
Age groups	20-30 yrs	12	43
	30-40 yrs	7	25
	40-50 yrs	5	18
	50-60 yrs	4	14
Ethnicity	IT	5	18
	FID	23	82
Classification of DP	Dental officers	12	43
	Dental technicians	16	57
Sector	Public/government	22	79
	Private	6	21
Division	Northern	7	25
	Western	5	18
	Central	16	57

**Table 4:** Themes and subthemes identified for FGD analysis.

Themes	Subthemes
CDP guidelines	CDP fabrication guidelines and clinical practice guidelines (CPG)
	DPs knowledge on CDP
Post-denture insertion advice	Guide and instruction to CDP wearing and care
	Patient motivation
CDP care and maintenance	Dos and don'ts of CDP care and maintenance
	Home care remedies to CDP care and maintenance
Challenges while treating EDPs	Language barriers
	Patient noncompliance
	CDP comparison (old CDP vs new CDP and patient to patient comparison)
Management strategies on challenges faced	Modifying CDP treatment and fabrication approach to meet patient needs
	Addressing of patient expectations from day 1 of treatment
	Promote effective patient participation throughout the treatment process
	Incorporating verbal, written, and translated advice to EDPs on their CDP
Practice of communication and teamwork	Staff communication-dentist and dental technician
	Triangle of communication and information sharing (dentist-dental technician and patient communication)
Recommendations to improving the quality of CDP delivery in Fiji	Further education for DPs
	Standardizing workload for DPs
	Decentralization of dental prosthetic services
	Increasing employability for DPs in CDP delivery

## Data Availability

The datasets used and/or analyzed during the current study are available from the corresponding author on reasonable request.
